# Improved Handover Authentication in Fifth-Generation Communication Networks Using Fuzzy Evolutionary Optimisation with Nanocore Elements in Mobile Healthcare Applications

**DOI:** 10.1155/2022/2500377

**Published:** 2022-01-07

**Authors:** J. Divakaran, S. K. Prashanth, Gouse Baig Mohammad, Dr Shitharth, Sachi Nandan Mohanty, C. Arvind, K. Srihari, Yasir Abdullah R., Venkatesa Prabhu Sundramurthy

**Affiliations:** ^1^Department of Electronics and Communication Engineering, K S R Institute for Engineering and Technology, Tiruchengode, Tamilnadu, India; ^2^Vardhaman College of Engineering, Hyderabad, India; ^3^Department of Computer Science and Engineering, Vardhaman College of Engineering, Hyderabad, India; ^4^Kebri Dehar University, Department of Computer Science and Engineering, Kebri Dehar, Ethiopia; ^5^Department of Electronics and Communication Engineering, Karpagam College of Engineering, Coimbatore, India; ^6^Department of Computer Science Engineering, SNS College of Technology, Coimbatore, India; ^7^CSBS, Sri Krishna College of Engineering and Technology, Coimbatore, India; ^8^Department of Chemical Engineering, Addis Abada Science and Technology University, Addis Ababa, Ethiopia

## Abstract

Authentication is a suitable form of restricting the network from different types of attacks, especially in case of fifth-generation telecommunication networks, especially in healthcare applications. The handover and authentication mechanism are one such type that enables mitigation of attacks in health-related services. In this paper, we model an evolutionary model that uses a fuzzy evolutionary model in maintaining the handover and key management to improve the performance of authentication in nanocore technology-based 5G networks. The model is designed in such a way that it minimizes the delays and complexity while authenticating the networks in 5G networks. The attacks are mitigated using an evolutionary model when it is trained with the relevant attack datasets, and the model is validated to mitigate the attacks. The simulation is conducted to test the efficacy of the model, and the results of simulation show that the proposed method is effective in improving the handling and authentication and mitigation against various types of attacks in mobile health applications.

## 1. Introduction

In recent times, the mobile and telecommunication devices get faster and more functional with each wireless network applicable on mobile health programs in healthcare. The speeds we have today were made possible by 4G [1]. Nevertheless, 4G networks are nearing their capacity limit as more people get online and demand even more data from their gadgets and smartphones. The researchers are now on the verge of transitioning to 5G, the wireless technology.

The increased traffic can be handled on this network than on Long-Term Evolution (LTE) networks. The 5G mobile network concept is being discussed by both business and academia. Next-generation mobile networks should be in place by 2020, according to current estimates. With increasing data traffic, devices are being studied to see if it is possible to attain 1 ms latency [2]. There will also be new features in 5G, such as the heterogeneous network integration with the network security over reliability and provisioning [3, 4].

As a result of these performance requirements, various 5G network technology solutions have been implemented, including HetNets, software-defined networking (SDN), and more. SDN has gotten a lot of interest recently as a promising new technology for the next generation of wireless mobile networks [5–8]. Control plane and data forwarding are separated or decoupled in an SDN, allowing a centralised controller to take control of the network. The control plane of an SDN network is independent of data forwarding and programmable. This SDN functionality makes network configuration and reconfiguration much simpler [9].

Additionally, it offers excellent security management over network opportunities in terms of adaptability and programmability. In contrast, developing SDN and NFV technologies may run and instantiate networks and their services in order to minimise costs and improve performance [10]. The 5G heterogeneous networks are critical to achieving goals such as low energy consumption, low cost, and full coverage. HetNet heterogeneity allows for more coverage, higher capacity, and improved performance.

Different 5G cells, including relays, microcells, and femtocells are being proposed to support imminent coverage [11]. As a result, the next-generation network is expected to be significantly more heterogeneous, and because of the densified deployment of a small cell, users should expect to see more frequent handoffs [12–21].

Vertical handover is critical in such a heterogeneous environment because it allows different networks to be integrated with one another. As a result, the researchers will be able to take advantage of the best features of existing networks. For a registered and valid user to gain access to network resources, authentication is necessary. Furthermore, mutual authentication can maintain secrecy by protecting communication entities from diverse threats and ensuring the integrity of their data. Due to frequent user movement across multiple networks, a smooth and secure solution for handover authentication is required to protect against various attacks.

In order to provide secured access to users on a foreign network, a rapid and effective authentication mechanism must be designed. However, there are not many studies looking specifically at 5G mobile network architecture and security in mobile healthcare applications.

Due to certificate-based authentication high security and ability to provide authentication, a system based on shared key distribution for certificate authentication is proposed. Thus, users in the 5G network environment can be certified by other networks. It is intended that the effectiveness of security management techniques, as well as the overall network view, will be improved using an evolutionary model. Transport Layer Security (TLS) is used in the proposed approach, but it is enhanced with preinitial authentication, which gives a shared certificate to registered user equipment only. As a result, the suggested system incorporates mutual authentication, key exchange, and agreement components. Data integrity and privacy are also provided as well as resistance against many forms of attacks.

The main contributions are given as follows:

- Using the SDN for network management and security, as well as the HAU for seamless and effective handover, helps to create a global perspective of the network.
- To provide great security and mutual authentication, the TLS protocol should be used.
- This ensures that vertical handover processes are consistent and secure because the certificate authentication relies on key distribution that has a fuzzy evolutionary model. The evolutionary model maintains the handover and key management to improve the performance of authentication with nanocore elements in 5G networks.

## 2. Related Works

By extending the 3GPP LTE hierarchical architecture and integrating the SDN technology, they presented a 5G mobile network architecture that can leverage intelligence and programmable networking capabilities. An authentication handover [22] based on SDN functions is presented in the design, and this allows subscribers to track their movements and their next location to be monitored. As a result, AHM is able to recognise prospective target cells and begin the handover operation to minimise the associated signalling delay.

Symmetric key cryptography and Elliptic Curve Diffie–Hellman are used in [23] to propose an authentication mechanism for LTE networks. With the addition of a local authenticator, they fixed the flaws in the EAP-AKA protocol. As a result, this approach can safeguard user identification against a variety of attacks while also enabling data integrity and mutual authentication across users. In the context of 5G networks, the approach may not be efficient or scalable due to the high number of small cells and users.

He et al. [24] presented a technique based on binary pairing functions to secure the operation of handover and reduce the communication and computation costs as an alternative authentication scheme. The delay can be as high because the authentication server is normally placed remotely, which makes it unsuitable for 5G requirements due to frequent handovers between the authentication server and tiny cell access points.

An evolved packet system in LTE networks was proposed by in [25] to overcome numerous flaws of EAP by lowering computational overhead and authentication latency and satisfying security requirements. EPS uses simple password key exchange. With a secret key, the major goal is to keep the user UE private while also minimising the size of sent messages and speeding up the protocol. The authentication process gets more simplified, but there is a risk of increased delays in 5G small cell networks due to a higher frequency of enquiries.

## 3. System Model

In order to have robust security against multiple attacks, the heterogeneous 5G mobile network environment should match the criteria of secured data transmission from mobile health applications [26, 27].

The researchers also need to meet the following requirements: mutual authentication, data privacy and integrity, and protection from passive and active attacks such as DoS and Man in the Middle (MitM) attacks. Because millimetre waves have poor signal transmission characteristics and operate at very high frequencies, the 5G mobile network is more heterogeneous, with many tiny cells.

Network accessing over UE differs from that of access points (APs) and evolved network nodes (eNBs). Using 5G multilayer coverage, this heterogeneous paradigm not only keeps up with the progress of existing technologies but also meets the data traffic demand with small cells that provide extremely high throughput and underlying macrocells that provide ubiquitous coverage even with small cell deployment. Minimal power tiny cells are, therefore, expected to be a significant part of the 5G network, enabling users to communicate at low cost while also providing great capacity.

Figure 1 shows the handover authentication unit (HAU) installed in the 5G mobile network SDN controller, which underpins SDN technology.

All 5G access points, base station (BS), and switches are equipped with relevant SDN protocols to support SDN-enabled 5G networks. To ensure flawless handover authentication, the implemented HAU must keep tabs on and forecast the locations of registered mobile users and then prepare the necessary BS and APs before the users arrive. The HAU stores and analyses user data by employing a traffic flow filter to collect physical layer attributes from registered users. Once user equipment has been preauthenticated for the first time, data collection will begin.

The study uses a downlink LTE system, where the eNB is placed within the UE (*u*) set. It is then distributed inside the network coverage range. The eNBand UE is of a single SISO antenna type.

We consider the user set *S* = {1, 2,…, *S*} with the service set *u*_*s*_, where ∪_*s*∈*S*_*u*_*s*_=*u* and *s* ∈ *S*. Each individual user is allowed to authenticate the network for one time ∩_*s*∈*S*_*u*_*s*_=∅.

While TDMA is employed in LTE, the OFDMA technology is used in the multiple access strategy. Due to signalling limits and the assignment of radio resource blocks, this is taken into account. The LTE system places the K RBs in *k* sets, which are then distributed. The TTI is the period of time during which the UE is given access to the RRA algorithm-allocated resources. The TTI here is the same as the RB timing duration, and each RB is assigned to a single UE for the period of a single TTI.

Each TTI complex channel coefficient *h*_*u,k*_ contains the propagation effects over the LTE channel, such as shadowing, path loss, and small-scale fading UE (*u* ∈ *U*) and eNB over RB (*k* ∈ *K*). Channel response is referred to as a complex channel coefficient because coherence is greater than RB; hence, the channel fades flatly. Subcarrier and the 1st OFDM symbol are the most common uses for this. In order to estimate the *h*_*u,k*_, UE uses pilot symbols, and the data are transmitted via eNB for transmission. This estimates the channel ${\hat{h}}_{u,k}$ to be as, and it is modelled as follows:

(1) $$\begin{array}{c} {\hat{h}}_{u,k}=\sqrt{\left(1-\xi \right)h_{u,k}}+\sqrt{\xi_{\eta }}, \end{array}$$

where *ξ* ∈ (0, 1)- channel estimation degradation and *η*∈*C-* channel estimation error.

The channel estimation error is modelled as a random variable as follows:

(2) $$\begin{array}{c} E\left\{{\left|\eta \right|}^{2}\right\}=E\left\{{\left|h_{u,k}\right|}^{2}\right\}. \end{array}$$

The current research finds the authentication error linked to channel estimate errors, and the parameter *ξ* is assessed depending on the impact of those flaws. Finally, reports are taken into account at each TTI, and the eNB obtains measurements immediately.

Additionally, the estimated instantaneous SNR ${\hat{\gamma }}_{u,k}$ for each TTI is determined as follows:

(3) $$\begin{array}{c} {\hat{\gamma }}_{u,k}=\frac{p_{u,k}{\left|{\hat{h}}_{u,k}\right|}^{2}}{\sigma^{2}}, \end{array}$$

where *p*_*u,k*_- eNB power and *σ*^2^- AWGN power.

The link adaptation mechanism, which is employed in LTE as well, selects the MCS (*m*) from a list of MCSs using eNB (*M*).

When applied to the set, the MCS selection employs ${\hat{\gamma }}_{u,k}$ and considers *M* = |*M*| with varying MCS, where |·| specifies the cardinality. The UE *u* in *k-*related MCS *m*_*u,k*_ is determined as follows:

(4) $$\begin{array}{c} m_{u,k}=f\left({\hat{\gamma }}_{u,k}\right), \end{array}$$

where *f* (${\hat{\gamma }}_{u,k}$)- link adaptation function.

The eNB used in this study selects the superior MCS from among the available UE, resulting in a higher data rate per unit of network power consumed.

UE uses MCS to transmit information to the eNB, which assures the block error rate value. The needed block error rate value is utilised to acquire the link adaption curve with minimal SNR ${\hat{\gamma }}_{u,k,m}$, and it is evaluated as follows:

(5) $$\begin{array}{c} {\hat{\gamma }}_{u,k,m}=f^{-1}\left(m_{u,k}\right), \end{array}$$

where *f*^−1^(·)- inverse link adaptation function.

The throughput rate *r*_*u,k,m*_ over a user *k* of UE *u* through a multichannel system *m* is illustrated as follows:

(6) $$\begin{array}{c} R_{u}=\sum_{k=1}^{K=\left|K\right|}\sum_{m=1}^{M=\left|M\right|}r_{u,k,m}x_{u,k,m}, \end{array}$$

where *x*_*u,k,m*_- assignment allocation index.

The authentication *τ*_*u*_ for the UE *u* is obtained via *R*_*u*_ rate using *φ*(·) function as follows:

(7) $$\begin{array}{c} \tau_{u}=\phi \left(R_{u}\right). \end{array}$$

## 4. Proposed Method

Because the 5G mobile network will be highly heterogeneous, mutual authentication between the users and server is one network criterion. The suggested system makes use of mutual authentication and FEA-TLS security capabilities. Apart from these characteristics, FEA-TLS comes with even more noteworthy ones, including fragmentation, key exchange and agreement, reauthentication, and resilience to MitM and replay attacks.

When it comes to the FEA-TLS protocol specification, the following shows the process of the proposed protocol:

- Public key infrastructure is used by FEA-TLS; therefore, certificates are required
- The UE and the authentication server are the first points of contact
- The certification authority issues certificates to authentication servers and user equipment
- The user equipment certificate must be validated with a network server during the UE lifetime
- To verify a user certificate, the authentication server needs a certificate from a certification authority

### 4.1. Proposed FEA-TLS Protocol

According to the estimations, the suggested protocol is more efficient than other evolutionary TLS-based systems when it comes to handover authentication with the signed certificate. It also fits the 5G mobile network requirement for a heterogeneous environment. Key exchanges are made possible with the deployment of this FEA-TLS-based system for authenticating user equipment.

An initial authentication strategy using shared key cryptography is proposed for use in the new protocol, and this key will be utilised by the UE to obtain a certificate and gain access to resources on the foreign network during vertical handover. UE requests for the foreign network certificate rather than transferring it straight from that authority to UE, which is one of the key aspects of the proposed system.

Figure 2 shows the beginning of the handover authentication procedure.  Figure 3 shows the process as it continues. As a result, the proposed technique protects the UE identity from being attacked.

#### 4.1.1. Preinitial Authentication

The user equipment will transmit the handover request and physical layer attributes to the home network eNB. The HAU then verifies these data before distributing the symmetric keys. eNB on the home network then responds with symmetric keys from the home networks, as depicted in Figure 2.

#### 4.1.2. FEA-TLS Authentication

Before the UE begins the authentication process, the eNB shares the identity of UE with the AP of a foreign network for the identification verification process that is provided by the UE during the handover request, as illustrated in Figure 3. The UE will now send the AP a start packet. It is common for this AP to send the UE a FEA-TLS request packet. The UE responds to the AP with a packet including identification information.

As soon as the AP receives the UE identification information, it compares it with the UE id received from the eNB in the home network and confirms the information. Additionally, the AP will need to send an empty FEA-TLS/start packet, which is an FEA-TLS-packet type with the start bit set, to the UE during this verification process. The UE will send a welcome message with a cipher message, packet type, a session Id, and a random number to begin the FEA-TLS interaction.

This will be followed by a response from the AP with an EAP request packet with the FEA-TLS packet type along with the hello message and version number along with an acknowledgement to begin key exchange with the AP settings. To verify the certificate, the UE will send an already shared symmetric key along with a signed response from it. This packet is subsequently forwarded to the AP, which verifies and responds with the completed message containing the signed certificate and key of the response of UE authentication to the AP. After receiving the completion handshake message, the UE responds using a null message if the verification was successful. This session will come to an end when the AP responds with a success message.

Assume that the home network registers the UE with a SIM and a key is shared between the two networks. Therefore, when the UE leaves its home network and enters a foreign network, it must gain access to the foreign network. Both parties to the roaming agreement have signed it, as shown in Figure 3.

Public keys that are known by the UE, home network, and the foreign network tend to get shared between the networks via the proposed FEA-TLS authentication. A certificate issued by the certification body is also present on both networks. SDN controller HAU shares user identity with the foreign network AP prior authentication based on UE location.

By eliminating the need to communicate identity verification to the HAU, this AP can perform UE identity verification faster, allowing for seamless authentication handover for the UE. As soon as the UE returns to its home network, the HAU will see if the new UE it just added is in the list of previously registered ones. As long as the UE is on the list, HAU will have access to its own private network.

## 5. Security Verification

This section conducts both informal analyses as shown below.

### 5.1. Mutual Authentication

FEA-TLS provides mutual authentication between the HAU and UE. With a handover request, the UE challenges the HAU preinitial authentication. Only the HAU has access to UE secret key, which grants UE network access.

### 5.2. User Identity Protection

The UE will have access to foreign Aps, if it requests a certificate. By distributing certificates in a fresh order, random variable, time, and the UE location are obscured. Each time a new user registers, the generation of temporary Id is carried out using a randomly generated variable. Aside from that, this temporary identifier will be altered at random, making it impossible to track down the original registrant. HAU in SDN has access to the user current location. By doing this, the user equipment identity is protected.

### 5.3. Signaling Overhead

In the FEA-TLS approach, authentication takes place between an AP of a foreign network and a user. Due to the SDN-enabled 5G network, there are no additional user ID verification and round-trip delays, and it takes much less time.

### 5.4. Passive Attack

A valid request packet may be obtained with this technique, but the message cannot be decrypted without private key. The fact that SHA-1 features a mechanism for generating keys makes it difficult to decrypt without the private key. As a result, the study designed the evolutionary system to be resistant to a passive attack.

### 5.5. MitM Attack

MitM attacks will not be able to succeed against this model. When an identity of the user is secured by a temporary public key pair issued by the UE, attackers cannot get their hands on or change the key, and thus, it is useless to them. As a result, the HAU only shares the UE identification with the AP when the UE makes a handover request and finds the UE position. As a result, passive attacks are not a problem.

## 6. Results and Discussion

In this section, the performance evaluation is conducted on fuzzy evolutionary algorithm to control the HAU. The model is compared with existing methods in terms of various metrics including space complexity, communication overheads, executed handovers, and latency in handover.

### 6.1. Communication Overheads

Figure 4 shows the communication overhead between FEA-TLS on HAU with existing fuzzy and TLS methods. The results of communication overhead show that the proposed FEA-TLS achieves reduced communication overhead than the other methods.

### 6.2. Space Complexities

Figure 5 shows the space complexity between FEA-TLS on HAU with existing fuzzy and TLS methods. The results of space complexity show that the proposed FEA-TLS achieves reduced space complexity than the other methods.

### 6.3. Handover Latencies

Figure 6 shows the handover latencies between FEA-TLS on HAU with existing fuzzy and TLS methods. The results of handover latency show that the proposed FEA-TLS achieves reduced handover latency than the other methods.

### 6.4. Executed Handovers

Figure 7 shows the executed handover between FEA-TLS on HAU with existing fuzzy and TLS methods. The results of executed handover show that the proposed FEA-TLS achieves highly successful handover than the other methods.

From the results, it cloud be inferred that the proposed method achieves higher rate of accuracy in detecting the attacks while the data are transmitted from mobile health programs in healthcare. This shows higher efficacy in improving the mitigation of attacks in the healthcare field.

## 7. Conclusions

In this paper, we proposed the fuzzy evolutionary model for handover and key management in 5G networks for improving the network performance in terms of authentication in mobile health programs. The use of nanocore elements in 5G hardware with the fuzzy evolutionary model reduces the computational complexity and delays while authenticating the messages and users. The evolutionary model mitigates the attacks during the training process with relevant datasets, and the validation shows improved detection accuracy for the mitigation of the attacks. The simulation shows an improved efficacy of the fuzzy evolutionary model in terms of improved accuracy, and furthermore, it shows secured authentication of input messages and users into the network against various type of attacks in mobile health programs. The space complexity, handover latency, and executed handovers are minimal in the fuzzy evolutionary model than in other methods.

## Figures and Tables

**Figure 1:** Simplified 5G network architecture with SDN for medical datasets.

**Figure 2:** Healthcare security (initial authentication).

**Figure 3:** Flow of authentication for medical data.

**Figure 4:** Communication overhead in the medical database.

**Figure 5:** Space complexity for medical databases.

**Figure 6:** Handover latency in patients' history.

**Figure 7:** Executed handover security in the medical Mongo database.

## Data Availability

The datasets used and/or analyzed during the current study are available from the corresponding author on reasonable request.
